# Effects of Nano-particles on Histo-pathological changes of the fish

**DOI:** 10.1186/s40201-015-0216-9

**Published:** 2015-08-29

**Authors:** Ali Louei Monfared, Ali Mohammad Bahrami, Ehsan Hosseini, Salman Soltani, Minoo Shaddel

**Affiliations:** Faculty of Para-Veterinary Medicine, University of Ilam, Ilam, Iran; Master of Sciences of Histology, Faculty of Veterinary Medicine, University of Shahid Chamran Ahwaz, Ahwaz, Iran; Department of Parasitology, Faculty of Medicine, Aja University of Medical Sciences, Tehran, Iran

**Keywords:** Biochemistry, Carp, Gill, Histology, Kidney, Nanosilver

## Abstract

Regarding fast development of the nanotechnology and the probably of it’s side effects on aquatic body organs, this study investigate the effects of nanosilver administration on histology of gill, kidney and biochemical parameters in common carp. The silver nanoparticles were synthesized in a one-step reduction process in an aqueous solution. 60 O. mykiss were obtained from a local commercial hatchery. Fish were divided randomly into four groups. Control group was kept in dechlorinated tap water without any add-on material. Experimental groups were exposed to concentration of 3, 300 and 1000 mg/L of nanosilver solution for eight weeks, respectively. Biochemical analyses of sera, histological alterations of the gill and kidney tissue were done. Aneurism in the secondary lamellae and hyperplasia of epithelium in gills, adhesion of the gill lamellae, inducing hyaline cast formation, significant decreasing in the glomerular diameter and formation of intra cytoplasmic vacuoles in the various urinary tubules were seen in experimental groups. The serum levels of total protein was decreased significantly (*P* < 0.05) by increasing nanosilver concentration but ALP, LDH, AST and ALT increased significantly (*P* < 0.05). It is concluded that nanosilver induces gill and kidney damages and changes the biochemical parameters of O. mykiss juveniles in different concentrations.

## Introduction

Recently, a vast variety of nanomaterials have been developed and nanotechnology has emerged as rewarding key research area in the modern scientific set-up. It is the science of nanoparticles that show new and different properties compared to what they exhibit on a macroscale, enabling unique applications [1]. Due to the wide application of nanomaterials in industry, agriculture, business, medicine and public health; nanotechnology has gained a great deal of public interest [2].

Silver found in the body of mammals (including humans) has no known biological purpose and is suspected of being a contaminant [3]. Silver, as ionic Ag+, is one of the most toxic metals known to aquatic organisms in laboratory testing, although large industrial losses to the aquatic environment are probably infrequent because of it’s economic value as a recoverable resource [4]. Silver, however, is of concern in various aquatic ecosystems because of the severity of silver contamination in the water column, sediments, and biota.

Long-term industrial or medical exposure to silver and it’s compounds may increase blood concentrations of silver to levels which can have toxic effects, such as induction of sarcomas, anemia, and enlargement of the heart [5]. It has been reported the toxicity of silver nanoparticles in zebrafish models. Their results suggest that silver nanoparticles induce a dose-dependent toxicity in embryos, which hinders normal development [6]. In fish and amphibian toxicity tests with 22 metals and metalloids, silver was the most toxic tested element as judged by acute LC50 values [7].

Regarding fast development of the nanotechnology and it’s diverse applications, is very important having enough data on the probably it’s side effects on the aquatic body organs. Therefore, these studies investigate the effects of nanosilver administration on histology of gill and kidney biochemical parameters in common carp.

## Materials and methods

The silver Nanoparticles (Ag-NPs, were purchased from nanonasb pars, Tehran- Iran) were synthesized in a one-step reduction process in an aqueous solution. In a typical preparation, a 400-μL aliquot of a 0.1-M AgNO3 aqueous solution was added into 100 mL of an aqueous solution containing 0.10 wt. % of the soluble starch and vigorously stirred for 1 h. The pH of the resulting solution was adjusted to 8.0 by adding 0.1 M NaOH solution. Under this experimental condition, the initial reaction mixture was colorless, and the growth of the AgNPs was monitored at different intervals using UV-vis absorption spectroscopy. After about 1 h, the solution turned light yellow, which indicated the initial formation of the AgNPs. The mixture was maintained at 50 °C for 24 h, and the color of the reaction solution became yellow.

Sixty *O. mykiss* (weight = 130 ± 6.9 g; Total length = 11.52 ± 2.5 cm) were obtained from a local commercial hatchery (Ilam, Iran). Fish were transported in well aerated condition to the laboratory of freshwater fish research station in Ilam University. They were kept for a week in 200 L aquariums to acclimatize to the laboratory environment. During this period, they were fed five times a day (at 08.00, 11.00, 13.00, 15.00 and 18.00 h) by commercial pellets (33 % protein). After acclimatization, they were divided randomly into four groups. Control group was kept in dechlorinated tap water without any add-on material, while experimental groups were exposed to concentration of 3, 300 and 1000 mg/L of nanosilver solution, respectively for eight weeks (The doses in the present paper were selected based on the preliminary study as a pilot work). Each treatment was done in two replicates. The water was renewed every 12 h as 30 % of nanosilver is lost by volatilization [8]. At the end of the experiment, the fish were weighted, sacrificed and blood samples were collected by cardiac puncture. All of the procedures were carried out in accordance with institutional guidelines for animal care and use. In order to study morphological aspects, first the total length and body weight were recorded, and then the gill and kidney was removed from body to be weighed and measured. Condition factor (CF) for each fish were calculated according to following standard formula:

$$ \mathrm{C}\mathrm{F} = \mathrm{body}\ \mathrm{weight}\ \left(\mathrm{g}\right)/\mathrm{fork}\ {\mathrm{length}}^3\left(\mathrm{cm}\right) \times 100 $$

For histological evaluation, gill and kidney samples were taken and washed with saline. The samples fixed in buffered formalin (10 %), processed for sectioning (5-6 μm) and stained with H&E. The sections were examined with an Olympus BX60 microscope and visualized through the Color-View Camera (Olympus, Tokyo, Japan).

For biochemical assaying, the blood samples were centrifuged (5 min at 5000 g, Hettich D7200) immediately at room temperature and plasma were separated and stored at −20 °C until analysis. Total protein and albumin were assayed by biuret and Bromocresol green binding method, separately (ZiestChemie, Iran). Glucose was determined through the glucose oxidase method (ZiestChemie, Iran). Serum value of Total cholesterol was assayed by enzymatic-colorimetric method (ZiestChemie, Iran). Lactate dehydrogenase (LDH), Alanine aminotransferase (ALT), aspartate aminotransferase (AST) and alkaline phosphatase (ALP) were measured by kinetic enzyme assays (ZiestChemie, Iran). All data are presented as mean ± SD. Data were analyzed by one-way ANOVA followed by Duncan’s multiple comparisons test. Multiple comparisons tests were only applied when a significant difference was determined in the ANOVA analysis, *P* < 0.05. The SPSS 13.0 (Chicago, USA) was used for analyzing the results.

## Results

No mortality was recorded during the period of study in experimental and control groups. Fish exposed to different concentration of nanosilver for 8 weeks showed significant reduction (*P* < 0.05) in the renal weight and CF ratio compared to control group (Table 1). In the nanosilver exposed fish kidney weight and also CF ratio has been showed a significant decreasing when compared to control fish (Table 1). Furthermore, the tissue of gill and kidney findings from nanosilver exposed fish are illustrated in Fig. 1. In the control group, the gill and kidney exhibited a normal architecture and pathological abnormalities were not seen. In the gill tissues of the exposed fish to nanosilver; aneurism in the secondary lamellae of gills, hyperplasia of epithelium of gills as well as the adhesion of the gill lamellae were seen, as compared with control animals (Fig. 1a, b, c). In addition, treating with silver nanosilver could induce hyaline cast formation, significant decreasing in the glomerular diameter and also formation of intra cytoplasmic vacuoles in the various urinary tubules (Fig. 1d, e, f) (Table 2).

**Table 1:** Some morphometric measurments (means ± SD) in control and treated common carp (*Cyprinus carpio* )with different concentrations of nanosilver particles

Parameters/Groups	Control	3 mg/L of nanosilver particles	300 mg/L of nanosilver particles	1000 mg/L of nanosilver particles
Renal weight(g)	1.47 ± 0.16	0. 97 ± 0.12	1.03 ± 0.16	0.98 ± 0.09
Condition Factor (CF)	1.74 ± 0.03 ^a^	0.90 ± 0.05 ^b^	1.15 ± 0.05 ^b^	0.96 ± 0.29 ^b^

* Means in the same row with different letters are significantly different (ANOVA, *P* < 0.05)

**Fig. 1:** **a** Transverse section through the gill of the 3 mg/L of silver nanosilver treated fish. The figure shows the aneurism in the secondary lamellae of gills (arrow). (Haematoxylin and Eosine stain) (×400). **b** Transverse sections through the gill of the 300 mg/L silver nanosilver treated fish. The figure shows the hyperplasia of epithelium of gills (arrow). (Haematoxylin and Eosine stain) (×400). **c** Transverse sections through the gill of the 1000 mg/L silver nanosilver treated fish. The figure shows adhesion of the gill's secondary lamellae (arrow). (Haematoxylin and Eosine stain) (×400). **d** Transverse sections through the renal tissue of the 3 mg/L silver nanosilver treated fish. The figure shows hyaline cast formation (arrow) in the lumen of the proximal convoluted tubules of kidney. (Haematoxylin and Eosine stain) (×400). **e** Transverse sections through the renal tissue of the 3 mg/L silver nanosilver treated fish. The figure shows a significant decreasing in the glomerular diameter (arrow) in the kidney of nanosilver administrated fish. (Haematoxylin and Eosine stain) (×400). **f** Transverse sections through the renal tissue of the 3 mg/L silver nanosilver treated fish. The figure shows the formation of intra cytoplasmic vacuoles in the various urinary tubules (arrow) of the kidney. (Haematoxylin and Eosine stain) (×400)

**Table 2:** Some histometric indices (means ± SD) in control and treated common carp (*Cyprinus carpio*) with different concentrations of nanosilver particles

Parameters/Groups	Control	3 mg/L of nanosilver particles	300 mg/L of nanosilver particles	1000 mg/L of nanosilver particles
Diameters of renal corpuscle (μm)	689.9 ± 11.5 ^a^	455.2 ± 7.85 ^b^	345.3 ± 4.67 ^b^	231.1 ± 11.2 ^b^*
Diameters of lumen of proximal convoluted tubules (μm)	4.96 ± 0.07 ^a^	7.1 ± 0.05 ^b^	7.3 ± 0.05 ^b^	7.7 ± 0.03 ^b^
The height of epithelium of proximal convoluted tubules (μm)	29.9 ± 0.03 ^a^	17.4 ± 0.05 ^a^	18.3 ± 0.05 ^a^	17.6 ± 0.08 ^a^

*Means in the same row with different letters are significantly different (ANOVA, *P* < 0.05)

The serum levels of total protein was decreased significantly (*P* < 0.05) by increasing nanosilver concentration. Other parameters such as ALP, LDH, AST and ALT levels in sera of nanosilver treated fish showed a significant increase compare to the control group (*P* < 0.05) (Table 3). A dose dependency was recorded in measured parameters as increase in nanosilver concentration caused a significant change in all assayed parameters (*P* < 0.05).

**Table 3:** Some serum biochemical parameters (means ± SD) in control and treated common carp (*Cyprinus carpio*) with different concentrations of nanosilver particles

Parameters/Groups	Control	3 mg/L of phenol	300 mg/L of phenol	1000 mg/L of phenol
Total protein(g/dl)	4.66 ± 0.47 ^a^	2.58 ± 0.21 ^b^	2.14 ± 0.34 ^b^	3.03 ± 0.67 ^b^
Albumin(g/dl)	3.8 ± 0.08 ^a^	3.67 ± 0.09 ^a^	3.78 ± 0.03 ^a^	3.25 ± 0.03 ^a^
Total cholesterol (mg/dl)	100.6 ± 7.6 ^a^	100.6 ± 5.9 ^a^	101.0 ± 7.6 ^a^	108.1 ± 6.3 ^a^
Glucose(mg/dl)	72.3 ± 3.4 ^a^	71.9 ± 6.3 ^a^	72.4 ± 3.1 ^a^	72.3 ± 3.9 ^a^
ALP (U/L)	67.73 ± 2.36 ^a^	83.45 ± 6.9 ^b^	95.3 ± 4.3 ^b^	89.6 ± 3.91^b^
LDH(U/L)	165.6 ± 13.8 ^a^	279.9 ± 3.8 ^b^	278.0 ± 7.8 ^b^	239.8 ± 4.7 ^b^
AST (U/L)	25.6 ± 4.6 ^a^	39.5 ± 5.6 ^b^	49.5 ± 6.3 ^b^	53.6 ± 7.8 ^b^
ALT(U/L)	9.9 ± 1.7 ^a^	14.6 ± 7.1 ^b^	17.8 ± 2.08 ^b^	17.2 ± 7.8 ^b^

*Means in the same row with different letters are significantly different (ANOVA, *P* < 0.05)

## Discussion

In the present study, significant alterations in the kidney weight, body condition ratio and also the gill and kidney structures as well as blood biochemistry were observed following the exposure to nanosilver administration. Body condition ratio is an indicator of the overall fish condition; it reflects fish shape and energy reserves and has been used to evaluate fish stress [9]. Several studies have demonstrated that morphological indices, CF are potential indicator of toxicant effects, providing information on the ability of individual to tolerate chemical pollution or other kind of environmental stress [10, 11]. Some reports have demonstrated that CF has been declined in fish exposed to environmental pollutants [12]. In this study significant reduction in CF was observed in the nanosilver treated groups, which supports previous findings about nanosilver effects on *Oreochromis aureus* juveniles [13]. There are several studies which have shown similar histological changes in the gill and kidney of fish, resulting from exposure to different toxic chemicals [13–17].

The findings of the present work showed significant structural effects in the experimental fish when compared with control animals. These alterations could be driven from the fish excessive activity to respiration and also get rid of the toxicant from its body during the process of detoxification [14]. Biochemical results of the present work showed a significant decrease in the serum levels of main serum enzymes in the nanosilver exposed fish. The decreased levels of total protein in fish exposed to nanosilver suggest that the protein might be used as an alternative source of energy, due to high energy demand that induced by nanosilver intoxication as it shown in *Brycon cephalus* [8].

The significant enhanced LDH activity levels in the fish exposed to nanosilver may be reflect the increased rate of conversion of lactate to pyruvate and then to glucose as reported in other species [8, 13]. Otherwise, the elevated serum ALP activity in the present study could be due to nanosilver cytotoxicity. In this study exposure to nanosilver resulted in a significant increase in the activities of plasma AST and ALT compared to control group. This is in accordance with finding of Nemcsók and Benedeczky in rainbow trout [18]. AST and ALT are plasma non-functional enzymes which are normally localized within the cells of many organs including kidney. They are also considered as an important indicator in assessing kidney status [19, 20] and tissue injury or organ dysfunction [21]. The increase in ALP, AST, and ALT after nanosilver exposure was in accordance with histopathological findings. Therefore, the increase of these enzymes is an indicator of gill and kidney damage and thus otherwise alterations in the gill and kidney function.

Although there are not a absolute mechanism of action for nanosilver gill and kidney toxic histological alterations; but previous study hypotheses that silver nanoparticles can disrupts the Na^+^ ,Cl^-^ and H^+^ exchanges at the gills, which initiates a complex chain of events culminating in cardiovascular collapse thereby insufficiency of gills in acting normal functions [22].

## Conclusion

This study showed that nanosilver induces gill and kidney damage and changes in serum biochemical parameters of *Cyprinus carpio* juveniles in different concentrations.
